The article "COVID-19 and Liver Dysfunction" was published in 2022. Journal: Cureus.

# COVID-19 and Liver Dysfunction

**DOI:** 10.7759/cureus.21302

**Published:** 2022-01-16

**Authors:** Nour Ibrahim, Jad Hosri, Yara Bteich, Alfred Dib, Antoine Abou Rached

**Affiliations:** 1 General Medicine, Faculty of Medical Sciences, Lebanese University, Beirut, LBN; 2 Department of Critical Care Medicine, Sacre-Coeur Hospital, Beirut, LBN; 3 Internal Medicine - Gastroenterology, Faculty of Medical Sciences, Lebanese University, Beirut, LBN

**Keywords:** coronavirus, liver function tests, hepatotoxic, cholestatic, hepatocellular

## Abstract

Introduction

The pandemic of coronavirus disease 2019 (COVID-19) has caused over four million deaths, depleting resources and healthcare workers; therefore, in an attempt to stratify patients, the relationship between liver enzymes and clinical outcome was studied. This study aimed to assess the pattern and impact of liver enzymes on the clinical outcome of hospitalized patients with COVID-19 in Lebanon and look for possible confounding factors.

Methodology

This was a single-centered retrospective cohort study conducted between December 2020 and March 2021 on 230 patients diagnosed with COVID-19. Liver function tests (LFTs) and other laboratory values on admission and peak hospitalization were analyzed using SPSS.

Results

The prevalence of abnormal liver tests among the sample population with severe COVID-19 infection were as follows: aspartate aminotransferase (AST), 77%; alanine aminotransferase (ALT), 49%; alkaline phosphatase (ALP), 12%; and gamma-glutamyl transferase (GGT), 37%. A severe COVID-19 infection was more likely present in patients with abnormal levels of AST (p = 0.015), ALP (p = 0.03), and GGT (p = 0.022). ANOVA test revealed no significant relationship between AST levels at peak hospitalization and the treatments received by the patient.

Conclusion

Abnormal liver function tests of patients at admission may be an indicator of more severe disease. In the context of scarce resources created by the pandemic, it becomes essential to establish a reliable predictor for a severe outcome of COVID-19 infection and manage accordingly.

## Introduction

Coronavirus disease 2019 (COVID-19) was declared a global pandemic by the World Health Organization (WHO) on March 11, 2020. Since then, it has caused over four million deaths while posing major challenges to the healthcare systems worldwide. In Lebanon, the virus remains a threat as it has caused over 500,000 cases (as of August 2021) with two major waves of the pandemic pushing healthcare systems and their resources into a state of disarray [1].

The severe acute respiratory syndrome coronavirus 2 (SARS-CoV-2) mainly targets the respiratory system, causing pneumonia with clinical features such as fever, fatigue, cough, and dyspnea; however, literature has shown that it is a systemic disease affecting the gastrointestinal, nervous, and hematologic systems [2,3].

Systemic inflammation is in part responsible for the multisystem involvement, while the direct entry of the virus into cells through the ACE-2 receptor is responsible for damage to systems with cells expressing this receptor. Interestingly, it is expressed not only on the surface of alveolar type 2 cells but also on cholangiocytes and hepatocytes [4]. Consequently, trends of elevated levels of liver enzymes in patients with COVID-19 prompted the study to their clinical significance, proving their use as predictors for severe outcomes [5]. This relationship has not yet been studied on patients in Lebanon, and certain limitations have not been addressed as it is still not known whether the liver impairment can be attributed to the direct effect of the virus, to the host’s immune response, to the use of hepatotoxic drugs, or to a combination of these factors. This study aims to assess the pattern (hepatocellular, cholestatic, and mixed) and impact of liver enzymes on the clinical outcomes of hospitalized patients with COVID-19 in Lebanon and look for possible confounding factors such as hepatotoxic drugs given in such a situation.

## Materials and methods

Patients and study design

This is a single-centered retrospective cohort study conducted between December 2020 and March 2021. Medical records of patients diagnosed with COVID-19 at Sacre-Coeur Hospital in Beirut, Lebanon, were reviewed. All 230 patients included in the study tested positive for COVID-19 by nasopharyngeal swab PCR, had radiological findings indicative of COVID-19 as shown by thoracic CT scan, and presented with at least one of the COVID-19 clinical manifestations (e.g., fever, cough, dyspnea, sore throat, malaise, muscle aches, anosmia, nausea, vomiting, and diarrhea). Subjects with liver comorbidities including hepatitis, cirrhosis, liver cancer or metastases, and chronic alcoholism were excluded from the study. Other exclusion criteria included patients less than 20 years of age and those with no liver function tests ordered during their hospital stay.

Data collection

From the medical records, several variables were collected, such as demographic data (age, sex, date of admission and discharge, and comorbidities), clinical data (date of positive PCR result, date of symptom onset, and staging of patients based on disease severity), laboratory values (mainly aspartate aminotransferase (AST), alanine aminotransferase (ALT), gamma-glutamyl transferase (GGT), alkaline phosphatase (ALP), complete blood count with differential (CBCD), C-reactive protein (CRP), lactate dehydrogenase (LDH), creatine phosphokinase (CPK), blood urea nitrogen (BUN), creatinine, D-dimer, ferritin, fibrinogen, and others), and radiological data (percentage of lung involvement present on thoracic CT scan). A number of patients had their liver function tests repeated during their hospital stay, and these were selected for analysis and compared with admission results. Abnormal liver function tests (LFTs) were classified into two groups, i.e., above upper limit of normal (ULN) and two times ULN, and divided into two patterns, i.e., cholestatic (GGT and ALP) and hepatocellular (ALT and AST). Three researchers independently reviewed the data to ensure the homogeneity of the collected information.

The study protocol was reviewed and approved by the institutional review board (IRB) of the hospital under the name “ethical committee of Sacre-Coeur Hospital” and conducted in accordance with the principles of the Declaration of Helsinki.

According to the World Health Organization, adults with COVID-19 infection can be classified into mild, moderate, or severe illnesses. The criteria of severity in an individual are defined as follows: (1) SpO_2_ < 94% on room air at sea level, (2) arterial partial pressure of oxygen to fraction of inspired oxygen (PaO_2_/FiO_2_) < 300 mm Hg, (3) respiratory frequency > 30 breaths/minute, and/or (4) lung infiltrates > 50% on chest imaging.

Treatment strategies

Since there are no definitive treatment guidelines for COVID-19, multiple options have been used at the hospital: (1) standard of care, (2) standard of care and remdesivir, and (3) standard of care and remdesivir with baricitinib.

Standard of care was defined as the nonspecific therapy against COVID-19 consisting of a combination of antibiotics, steroids (dexamethasone 6 mg), and a prophylactic dose of anticoagulant.

For patients suffering from desaturation on admission and requiring oxygen therapy, support was given according to severity: (1) nasal cannula face mask, (2) non-rebreather face mask, (3) high-flow oxygen, (4) double-source oxygenation, (5) BiPAP machine, and (6) invasive mechanical ventilation (intubation).

The patient’s final outcome was classified as either discharged home or deceased.

Statistical analysis

Data entry and statistical analyses were conducted using IBM SPSS Statistics for Windows version 26 (IBM Corp., Armonk, NY, USA). Descriptive statistics were presented as mean ± standard deviation for continuous variables and as frequencies and percentages for categorical variables. Normality of distribution was assessed using graphical plots; chi-square and Fisher’s exact tests were used to evaluate the relationship between categorical variables. Paired sample t-test was used to evaluate the difference in the levels of biomarkers on admission and at peak hospitalization. Univariate and multivariable regression analyses were performed to determine the factors and predictors of severe COVID-19 infection. The level of significance was set at α = 0.05.

## Results

Of the 230 patients, the mean age was 60.16 ± 16.15 years, 68% were females, and 30.4% had no chronic comorbidities. The prevalence of abnormal liver tests among the sample population with severe COVID-19 infection were as follows: AST, 77%; ALT, 49%; ALP, 12%; and GGT, 37%. A severe COVID-19 infection was more likely present in patients with abnormal levels of AST (p = 0.015), ALP (p = 0.03), and GGT (p = 0.022). Table 1 depicts the clinical characteristics of the studied population along with their liver function tests on hospital admission.

**Table 1:** Clinical characteristics of patients with COVID-19 infection with their liver function tests on hospital admission p: statistical significance; HTN: hypertension; DM: diabetes mellitus; DL: dyslipidemia; CAD: coronary artery disease; ALT: alanine aminotransferase; AST: aspartate aminotransferase; ALP: alkaline phosphatase; GGT: gamma-glutamyl transferase

Characteristic	Total (N = 230)	Non-severe COVID-19 (N = 117)	Severe COVID-19 (N = 113)	p-value
Mean ± standard deviation				
Age, years	60.16 ± 16.15	59.18 ± 15.99	60.88 ± 16.15	0.622
CT chest involvement, %	52.73 ± 18.94	40.15 ± 14.47	65.78 ± 12.12	<0.0001
Gender, N (%)				0.597
Female	157 (68)	78 (66.7)	79 (70)	
Male	73 (32)	39 (33.3)	34 (30)	
Comorbidities, N (%)				
Previously healthy	70 (30.4)	39 (33)	31 (27)	0.387
HTN	22 (9.6)	13 (11)	9 (8)	0.648
DM	14 (6.1)	8 (7)	6 (5)	0.784
DL	20 (8.7)	12 (10)	8 (7)	0.483
CAD	21 (9.1)	6 (5)	15 (13)	0.041
Asthma	6 (2.6)	2 (2)	4 (4)	0.446
HTN, DM, and DL	15 (6.5)	8 (7)	7 (6)	0.803
HTN and DM	20 (8.7)	8 (7)	12 (11)	0.36
Others	42 (18.3)	21 (18)	21 (19)	0.865
Liver function tests, N (%)				
ALT, U/L				
Normal	119 (52)	61 (53)	58 (51)	0.791
>ULN	72 (32)	36 (32)	36 (32)	0.964
>2 ULN	36 (16)	17 (15)	19 (17)	0.720
AST, U/L				
Normal	86 (39.5)	53 (49)	33 (30)	0.05
>ULN	99 (45.4)	40 (37)	59 (54)	0.015
>2 ULN	33 (15.1)	15 (14)	18 (16)	0.706
ALP, U/L				
Normal	197 (92)	103 (96)	94 (88)	0.04
>ULN	11 (5)	2 (2)	9 (8)	0.03
>2 ULN	6 (3)	2 (2)	4 (4)	0.408
GGT, U/L				
Normal	156 (70)	85 (77)	71 (63)	0.025
>ULN	44 (20)	15 (14)	29 (26)	0.022
>2 ULN	24 (10)	11 (9)	13 (11)	0.7

Paired sample t-test revealed a significantly higher level of abnormal AST and ALP on admission than at peak hospitalization (p = 0.001, difference of 12.97 ± 43.11 U/L, confidence interval (CI) = [5.31,20.63] and p = 0.014, difference of 12.80 ± 55.51 U/L, CI = [2.63,22.96], respectively), while none among the other liver tests. This was followed by a one-way ANOVA test that revealed no significant relationship between AST levels at peak hospitalization and the treatments (standard of care, standard of care and remdesivir, and standard of care and remdesivir with baricitinib) received by the patients. Deceased patients had significantly higher levels of neutrophils, urea, and LDH on admission and at peak hospitalization than those who recovered (Figure 1). On the other hand, lymphocytes and albumin were significantly higher in discharged patients than among deceased patients. Patients presenting with abnormal LFTs on presentation (at least one abnormal measure of ALT, AST, albumin, or total bilirubin) were at higher odds of having abnormal LFTs at peak hospitalization (crude odds ratio (OR) = 1.83, p = 0.035, CI = [1.042,3.208]). The predictors of AST levels in patients with COVID-19 at the time of peak hospitalization are summarized in Table 2, including age, LDH, neutrophils, and urea. The predictors of COVID-19 infection severity in patients on hospital admission and outcome at peak hospitalization are summarized in Table 3 and Table 4, respectively. The effect of treatment type of COVID-19 infection on the mortality of patients using logistic regression is presented in Table 5.

**Figure 1:** Marked differences in several laboratory indicators between deceased and discharged patients Death: gray Discharge: blue WBCs: white blood cells; LDH: lactate dehydrogenase

**Table 2:** Predictors of AST levels at the time of peak hospitalization in patients with COVID-19 p = 0.03; R2 = 0.66 B: beta value; OR: odds ratio; SE: standard error; p: statistical significance; CI: confidence interval Dependent variable: abnormal aspartate aminotransferase (AST) levels (normal AST levels (reference)); LDH: lactate dehydrogenase

	B	OR	SE	p-value	95% CI
Constant	-65.193	-1.904	34.243	0.089	[-142.655, 12.269]
Age	-0.647	-1.621	0.399	0.139	[-1.550, 0.256]
LDH	-0.145	-3.048	0.048	0.014	[-.252, -0.037]
Neutrophils	2.465	3.912	0.630	0.004	[1.040, 3.891]
Urea	0.336	1.570	0.214	0.151	[-0.148, 0.821]

**Table 3:** Predictors of severity of COVID-19 infection on admission B: beta value; SE: standard error; Wald: Wald test of true parameter; p: statistical significance; OR: odds ratio; CI: confidence interval Dependent variable: severe COVID-19 infection (non-severe COVID-19 infection (reference)) ALT: alanine aminotransferase; AST: aspartate aminotransferase; ALP: alkaline phosphatase; GGT: gamma-glutamyl transferase; WBCs: white blood cells; CAD: coronary artery disease; CPK: creatine phosphokinase; CK-MB: creatine kinase-myocardial band

	B	SE		Wald	P	OR	95% CI
Model 1							
Constant	-0.916	0.348		6.910	0.009	0.4	
ALT: on admission	-0.021	0.008		7.377	0.007	0.979	[0.964, 0.994]
AST: on admission	0.032	0.010		10.405	0.001	1.004	[1.013, 1.052]
ALP: on admission	0.001	0.002		0.051	0.821	1.001	[0.996, 1.005]
GGT: on admission	0.004	0.002		3.224	0.073	1.004	[1, 1.008]
Model 2							
Constant	-10.793		5.843	3.412	0.065	<0.0001	
WBCs: on admission	0.013		0.059	4.008	0.628	1.013	[0.962, 1.066]
Neutrophils: on admission	0.119		0.059	4.008	0.045	1.126	[1.003, 1.266]
Lymphocytes: on admission	0.079		0.069	1.310	0.252	1.083	[0.945, 1.240]
Model 3							
Constant	-0.605	0.301		4.030	0.045	0.546	
History of CAD reference: yes	1.626	0.671		5.872	0.015	5.081	[1.364, 18.922]
CPK: on admission	0.001	0.001		2.768	0.096	1.001	[1, 1.003]
CK-MB: on admission	0.011	0.015		0.510	0.475	1.011	[0.981, 1.041]
Troponin: on admission	0.001	0.001		0.410	0.522	1.001	[0.999, 1.002]

**Table 4:** Predictors of outcome of COVID-19 infection at peak hospitalization B: beta value; SE: standard error; Wald: Wald test of true parameter; p: statistical significance; OR: odds ratio; CI: confidence interval Dependent variable: outcome death (discharge (reference)) ALT: alanine aminotransferase; AST: aspartate aminotransferase; ALP: alkaline phosphatase; GGT: gamma-glutamyl transferase

	B	SE	Wald	P	OR	95% CI
Constant	-1.813	1.120	2.621	0.105	0.163	
ALT: at peak hospitalization	-0.087	0.039	5.077	0.024	0.916	[0.849, 0.989]
AST: at peak hospitalization	0.056	0.026	4.661	0.031	1.058	[1.005, 1.113]
ALP: at peak hospitalization	-0.003	0.007	0.164	0.686	0.997	[0.984, 1.010]
GGT: at peak hospitalization	0.002	0.008	0.056	0.813	1.002	[0.987, 1.017]

**Table 5:** Logistic regression model showing the effects of treatment types and other variables on the outcome of patients with COVID-19 infection B: beta value; SE: standard error; Wald: Wald test of true parameter; p: statistical significance; OR: odds ratio; CI: confidence interval Dependent variable: outcome death (discharge (reference))

	B	S.E.	Wald	P	OR	95% CI
Constant	-11.042	3.017	13.396	<0.0001	<0.0001	
Standard of care	-3.166	1.045	9.182	0.002	0.042	[0.005, 0.327]
Standard of care + Remdesivir	-1.306	1.279	1.043	0.307	0.271	[0.022, 3.322]
Standard of care + Remdesivir with Baricitinib	-1.670	0.943	3.137	0.077	0.188	[0.030, 1.195]
Age	0.152	0.042	13.244	<0.0001	1.164	[1.073, 1.264]
Sex Reference: Female	-1.446	0.717	4.070	0.044	0.236	[0.058, 0.960]

## Discussion

The present study illustrates that patients with severe COVID-19 infection had a higher incidence of abnormal liver function tests on admission and that the severity of infection was more likely associated with elevated levels of all LFTs except ALT. No particular comorbidity contributed to a worse outcome except for CAD, where 15 out of 21 patients (71.4%) had a severe infection. Not a single treatment strategy impacted LFTs, even days after the initiation of therapy. Higher levels of neutrophils, urea, and LDH prevailed in deceased rather than discharged patients. An increase in the levels of AST was attributed to severe COVID-19 infection and a higher mortality among patients. As for the predictors of abnormal AST at peak hospitalization, high neutrophils and LDH were most significantly correlated. The outcome of patients with COVID-19 infection was improved only in the sample of patients receiving standard of care regimen exclusively.

Our study aligns with previously published results confirming that elevated liver enzymes correlate with a more severe outcome [6-8]. The observed profile of liver function impairment was mainly mixed, i.e., both hepatocellular and cholestatic. Several proposed mechanisms for SARS-CoV-2-induced liver damage have been proposed: (1) systemic inflammation and cytokine storm [4], (2) direct cytopathic effect of the virus, and (3) hepatotoxic drugs. The last two mechanisms were part of this study’s interpretation. As highlighted by various studies, the entry of SARS-CoV-2 into the cells is primarily mediated by the binding of its S protein to ACE-2 receptors. ACE-2 receptors are expressed not only on alveolar type 2 cells but also on hepatocytes and cholangiocytes, a finding that can explain the previously mentioned mixed pattern of hepatic injury. However, the distribution of ACE-2 receptors on these cells is not proportional to cholangiocytes harboring the greater number [9]. Although this might intuitively lead to a predominant cholestatic pattern of liver injury, most studies observed either a predominant hepatocellular pattern or mixed pattern [5,9]. This can be explained by the fact that cholangiocytes have an important role in the regenerative capacity of the liver [4,10], the loss of which can be the reason for the hepatocellular damage. This discrepancy might indicate that the cytopathic effect of the virus may not be the main culprit for liver damage.

Within that hepatocellular pattern, AST levels were found to be higher than those of ALT. This disparity may be accountable to the presence of AST in tissues other than the liver, such as the heart, kidneys, skeletal muscles, brain, and RBCs, unlike ALT [11]. Therefore, injury to these organs or systemic inflammation, a finding not uncommon to COVID-19, can be responsible for the differential elevation of AST versus ALT, making ALT more specific for liver damage. Following this pattern of perturbation, direct liver damage from the virus is thus considered mild. This is also validated by the fact that mild elevation of these enzymes (less than two times ULN) was the only significant change observed. In addition, the different allocation of these enzymes with respect to hepatic acini, i.e., a higher concentration of AST in zone 3 [12], may present as a possible mechanism for the observed elevation of AST.

Remdesivir also plays a role in the pathogenesis of liver injury in the context of COVID-19 infection [13,14]. However, liver injury from the use of remdesivir (alone or with baricitinib) was not observed in our results. This may be due to the limited number of patients who received this treatment within the sample studied. Therefore, bigger sample size may be needed for a more definitive result. Nonetheless, experts suggest monitoring of liver enzymes during its administration.

The dynamic changes in LFTs observed between admission and peak hospitalization showed that AST and ALP were the highest on admission rather than later during the hospital stay. Multiple studies, however, discovered that the pattern of LFT evolution took a bell-shaped form [15,16], pertaining to increased levels throughout the patients’ hospitalization before normalizing at their discharge. These controversial findings likely relate to the unclear pathophysiology of COVID-19-induced liver injury and the different populations considered in the studies.

Besides disrupted LFTs, elevated LDH also served as a marker of severe outcome in COVID-19 disease, particularly resulting in a higher mortality rate. A study conducted by Li et al. confirmed this finding and stated that elevated serum LDH can be used to evaluate disease severity and predict in-hospital mortality in patients with COVID-19 infection [17]. In fact, LDH is an inflammatory marker released in response to hypoxia, cell death, and organ injury, all these processes being considered the main pathogenetic mechanisms of COVID-19 infection. Another relevant factor predicting mortality is blood urea nitrogen (BUN); this marker reflects a worse outcome in patients with heart failure and is a component of the CURB-65 score of community-acquired pneumonia [18]. This confirms BUN as a predictor of multiple organ failure and therefore a predictor of mortality from COVID-19 disease. One last parameter related to increased mortality is neutrophilia. Neutrophils constitute a major line of defense in innate immunity; however, unregulated production of pro-inflammatory cytokines exaggerates the immune response and worsens the initial offense. Neutrophilia also impairs the synthesis of nitric oxide, a proven antiviral agent, by decreasing the availability of arginine, which is an important substrate for NO synthesis [19].

Our results identified three major predictors positively correlated with a severe outcome from COVID-19 infection: elevated AST levels (both at admission and peak hospitalization), elevated neutrophil count (at admission), and the presence of CAD among other comorbidities (at admission). Despite the association between elevated cholestatic enzymes and severe infection, there does not seem to be a positive correlation between the two, meaning that GGT and ALP could be elevated without affecting the outcome of the patient. Interestingly, elevated ALT levels appeared to have a protective effect on patient outcomes. One speculative explanation behind this may be related to the more specific nature of ALT to liver inflammation, unlike AST, an enzyme commonly elevated as a response to the damage of other organs. This possibly postulates a greater impact of concomitant multiple organ damage on illness severity and patient outcome rather than liver involvement solely. Further research should target this hypothesis.

Regarding the optimal treatment regimen of COVID-19 infection, conflicting results are present regarding the superiority of remdesivir with or without baricitinib over dexamethasone alone [20]. Nevertheless, our findings revealed that an improved outcome was witnessed only among patients with COVID-19 infection who received standard of care. The findings to date are still inconclusive; thus, assessing the cost-effectiveness of different treatment modalities becomes indispensable, especially in developing countries where access to such drugs may be limited.

Among the several comorbidities, patients with CAD ended up developing a severe infection in the majority of cases. Multiple mechanisms may explain this association: (1) a strong correlation between coronary artery disease and viral infections (e.g., influenza), (2) direct viral invasion of the cardiac myocytes through the ACE-2 receptors, and (3) indirect immune response with increased levels of pro-inflammatory cytokines (TNF-alpha) [21]. However, several studies found that CAD is not an independent risk factor for mortality and severity in COVID-19 infection, as it was evidenced by the lack of significant correlation between CAD and complications such as ARDS, septic shock, and respiratory failure [21,22]. Moreover, the increase in the severity of illness in patients with CAD seen in our study may also be attributed to the prevalent use of ARBs and ACEI drugs among such patients due to the potential upregulation of ACE-2 receptors [23]. Nevertheless, a recent systematic review and meta-analyses revealed no significant difference in the illness severity of COVID-19 infection between ARB/ACEI users and nonusers [24]. Thus, future focus should be implemented on other comorbidities associated with CAD and their role in the mortality and severity of the infection while adjusting for other confounding variables.

Older age and male sex also contributed to a poor outcome. Marik et al. attributed this gender disparity to a heightened inflammatory response that occurs in men [25]. In fact, men express lower levels of ACE-2, resulting in higher levels of angiotensin II (promoting inflammation and oxidative stress) and lower levels of angiotensin I-7 (diminishing anti-inflammatory effects). Hence, this may explain why men have a greater risk of developing respiratory failure and severe inflammatory response compared with women.

Limitations

Our study has several limitations worth noting. This study was conducted in a single-center hospital in Lebanon with relatively small sample size, thus limiting its representativeness. As a retrospective study, not all liver enzymes were routinely ordered for all patients presenting with COVID-19 infection, accounting for missing data. Moreover, the time frame chosen for this study allowed for limited treatment strategies available for use to evaluate their impact on patient outcomes.

## Conclusions

In conclusion, patients with abnormal liver function tests at admission developed more severe disease. The pattern of disturbed LFTs was mixed (cholestatic and hepatocellular); however, only elevated AST levels correlated with a poorer outcome. This finding can further guide physicians to predict that outcome and provide more aggressive treatment when needed. Other predictors of severe disease were elevated neutrophil count and a history of CAD. Treatment strategies had no impact whatsoever on LFTs despite the recommendations to monitor them during the course of therapy. This calls for the conduction of larger studies involving a more representative sample of the population to better elucidate all the mechanisms behind liver injury in patients with COVID-19.
